The article "Fluorescence-guided surgery for cancer patients: a proof of concept study on human xenografts in mice and spontaneous tumors in pets" was published in 2017. Journal: Oncotarget.

# Fluorescence-guided surgery for cancer patients: a proof of concept study on human xenografts in mice and spontaneous tumors in pets

**DOI:** 10.18632/oncotarget.22728

**Published:** 2017-11-30

**Authors:** Eliane Mery, Muriel Golzio, Stephanie Guillermet, Didier Lanore, Augustin Le Naour, Benoît Thibault, Anne Françoise Tilkin-Mariamé, Elizabeth Bellard, Jean Pierre Delord, Denis Querleu, Gwenael Ferron, Bettina Couderc

**Affiliations:** ^1^ Institut Claudius Regaud –IUCT Oncopole, University Toulouse III, Toulouse, France; ^2^ Institut de Pharmacologie et de Biologie Structurale, Université de Toulouse, Toulouse, France; ^3^ Fluoptics SAS, Grenoble, France; ^4^ Clinique vétérinaire Alliance, Bordeaux, France

**Keywords:** tumor targeting, optical imaging, fluorescence-guided surgery, integrins, spontaneous animal models

## Abstract

Surgery is often the first treatment option for patients with cancer. Patient survival essentially depends on the completeness of tumor resection. This is a major challenge, particularly in cases of peritoneal carcinomatosis, where tumors are widely disseminated in the large peritoneal cavity. Any development to help surgeons visualize these residual cells would improve the completeness of the surgery. For non-disseminated tumors, imaging could be used to ensure that the tumor margins and the draining lymph nodes are free of tumor deposits.

Near-infrared fluorescence imaging has been shown to be one of the most convenient imaging modalities. Our aim was to evaluate the efficacy of a near-infrared fluorescent probe targeting the αvβ3 integrins (Angiostamp™) for intraoperative detection of tumors using the Fluobeam® device.

We determined whether different human tumor nodules from various origins could be detected in xenograft mouse models using both cancer cell lines and patient-derived tumor cells. We found that xenografts could be imaged by fluorescent staining irrespective of their integrin expression levels. This suggests imaging of the associated angiogenesis of the tumor and a broader potential utilization of Angiostamp™. We therefore performed a veterinary clinical trial in cats and dogs with local tumors or with spontaneous disseminated peritoneal carcinomatosis. Our results demonstrate that the probe can specifically visualize both breast and ovarian nodules, and suggest that Angiostamp™ is a powerful fluorescent contrast agent that could be used in both human and veterinary clinical trials for intraoperative detection of tumors.

## INTRODUCTION

In oncology, if tumor resection is feasible, surgery is often the first therapeutic option. For peritoneal carcinomatosis, which can occur in cases of colorectal or ovarian cancer or rare peritoneal disease, several retrospective studies demonstrate that patient survival essentially depends on the completeness of macroscopic tumor resection and on adjuvant chemotherapy [1, 2]. The current surgical standard for all peritoneal cancers is to achieve a CC0 resection according to the completeness of cytoreduction score (CC0: absence of visible residual disease), as complete cytoreductive surgery has been associated with improved survival [2, 3] [4, 5].

Unfortunately, peritoneal carcinomatous extensions, multifocal spread of the metastases, and close contact with vital organs often lead to incomplete tumor resection. In addition, smaller nodules are difficult to detect, whether preoperatively by computed tomography scans or magnetic resonance imaging (MRI), or visually during surgery.

Optimizing the extensiveness of cytoreductive surgery without collateral damage is still a major challenge [6]. For other cancers, such as breast cancers, sarcomas, and gliomas, improved imaging could help detect small tumor deposits surrounding the main tumor. Detecting these using real-time imaging could help ensure the completeness of tumor removal with adequate tumor margins. Importantly, patients who have had complete tumor resection derive the most benefit from chemotherapy treatment compared with those who have had incomplete resection, particularly for locally invasive tumors such as gliomas [7].

Ultimately, for potentially invasive cancers such as breast cancer, some of the draining lymph nodes will likely require removal to determine the extent of cancer involvement. There are long-term side effects of lymph node removal; being able to visualize cancer cells in lymph nodes during surgery would help to decide how many lymph nodes (such as the sentinel and draining lymph nodes) require removal, and could ultimately result in a reduction in the unnecessary removal of lymph nodes [8].

An intraoperative imaging method that allows surgeons to visualize nodules smaller than 1 cm would therefore be valuable in order to minimize residual disease. Advances in optical fluorescence imaging, and especially in intraoperative imaging devices associated with the generation of tumor–targeted contrast agents, can enhance the normal vision of surgeons [4, 6, 9, 10]. In addition to morphological changes and/or discoloration of the tissue that guide the surgeon, molecular imaging has the potential to provide additional biological information about the cancerous tissue at molecular and cellular levels [7].

Fluorescence imaging is based on materials that are optically active under near-infrared (NIR) wavelength excitations (700–1450 nm). NIR fluorescence imaging provides two key advantages for the detection of tumors that are found at a tissue depth of more than 1 cm and are smaller than 1 cm : low absorption of the tissue, and minimal autofluorescence in the NIR spectral bands. Therefore, the use of an exogenous chromophore improves the imaging contrast [4]. For example, molecular imaging with optical techniques can visualize tumors via fluorophore-conjugated probes targeting tumor markers, and may facilitate complete excision of tumors and tumor micromasses that are beyond the visual capacity of the naked eye [9]. Stummer et al. showed a clinical benefit for patients with glioma following removal of tumors using 5-aminolevulinic-acid (5-ALA)-induced fluorescence guidance, in terms of completeness of tumor removal and progression-free survival [10]. Prospective human research by Sturm et al. and Yoo et al. used targeted probe and fluorescence-guided surgery, respectively, for sentinel lymph node identification, lung segmentectomy, and cancer surgery [11, 12].

We have previously used the fact that tumors are highly vascular (due to neoangiogenesis) to investigate a fluorescent RAFT-(cRGD)4 tracer molecule (Angiostamp™) able to target the α_v_β_3_ integrins expressed on endothelial cells. NIR fluorescence was visualized using Fluobeam^®^, an open fluorescent imaging system that can be used in intraoperative conditions. In a preclinical setting, we showed that the use of Angiostamp™ combined with Fluobeam^®^ allowed the specific detection of residual tumor deposits and inframillimetric metastases derived from human ovarian adenocarcinomas [13]. Using the same approach, Dutour et al. compared the quality and sensitivity of tumor/metastasis margin delineation and tumor resection (in osteosarcomas) using intraoperative NIR imaging to those guided by preoperative imaging (i.e., MRI subsequently confirmed by histopathological analysis). They showed that intraoperative imaging is effective in improving primary tumor and lung metastasis excision [14]. Both studies showed that chemotherapy did not alter Angiostamp™ tumor-specific targeting, nor the sensitivity of tumor detection [13, 14]. Similar results have been described by Harlaar et al. for ovarian cancer [15]. Finally, Josserand et al. showed that fluorescence detection of metastatic nodules could be also used in combination with electrochemotherapy [16].

Here, we propose a generalized use of Angiostamp™-mediated fluorescence detection of different types of tumors. Review of the literature suggests that 25–50% of tumors are expected to express α_v_β_3_ integrins; this low proportion of integrin-expressing tumors means that, as yet, no dye for their detection has been developed for general use in the clinic. In the present work, we evaluated the ability of Angiostamp™ combined with Fluobeam^®^ to detect several tumor types, irrespective of their α_v_β_3_ integrin expression. Using genetically modified tumor cells injected into mice, we analyzed the fixation of the Angiostamp™ molecules in order to highlight the targeting of the neovessels. We further evaluated the kinetics of tumor labeling in mice, and performed a proof of concept trial in four pets (dogs and a cat) bearing spontaneous cancers. Indeed, the comparative oncology approach, specifically referring to the study of pets with spontaneous cancer, offers a potential solution to lingering questions about drugs and their accumulation in tumors. In addition to the similarities in drug metabolism, the large size of pet dogs and their naturally occurring, biologically heterogeneous malignancies allow the validation of new anticancer agents [17, 18]. Key features of this model system are that it allows investigations to be carried out in immune-competent, large animals (pet cats or dogs) with naturally occurring tumors, which confers advantages such as the presence of naturally syngeneic tumor-associated vasculature and stroma, tumor heterogeneity, and host immune responses [17, 18]. We showed that it was feasible to perform surgery using fluorescence-guided imaging on pets bearing different types of tumors (breast tumors, ovarian cancer, and cutaneous carcinoma) whether these were subcutaneous or peritoneal tumors. The technique is nontoxic, and animals were returned to their owners after tumor removal. This procedure allowed us to specifically detect tumor cells in organs, as well as in tumor margins and draining lymph nodes. It allows a more rapid surgical intervention compared to a procedure without fluorescence detection. As many common canine cancers are comparable to common human cancers in etiology, biological behavior, response to therapy, and overall outcome, the strategy could be applied soon in clinical trials in humans.

## RESULTS

### Detection of non-α_v_β_3_-expressing nodules in many tumor cell types

In our previous publication, we showed that all xenografts derived from ovarian adenocarcinoma biopsies of patients (patient-derived xenograft, PDX) could be visualized using Fluobeam^**®**^ after an injection of Angiostamp™ [19]. Nevertheless, a review of the literature revealed that only 50% of human ovarian tumors express α_v_β_3_ integrins. Therefore, we decided to evaluate whether α_v_β_3_-negative tumors were as fluorescent *in vivo* as α_v_β_3_-positive tumors (Figure 1). We injected tumor cells with differing integrin status from two groups of patients (four patients bearing α_v_β_3_-positive tumors and four patients bearing α_v_β_3_-negative tumors) into nude mice, allowed them to grow, and then visualized the tumors following Angiostamp™ injection. Both types of tumors could be visualized using Angiostamp™/Fluobeam^®^ (Figure 1). We quantified the emitted signals *in vivo* (Figure 1A and 1B), using as a background value the brightest part of the image adjacent to the tumor. From previous data [13], we determined that a value above 2 represented the specific fixation of the probe to a tumor nodule. Tumor nodules in both cases (from α_v_β_3_-positive patients and α_v_β_3_-negative patients) exhibited the same fluorescence intensities.

**Figure 1:** Angiostamp™ detects ovarian tumor nodules independently of the level of ɑ_v_β_3_ integrin expression **(A, B)** *In vivo* real-time fluorescence images of nodules from one ɑ_v_β_3_^+^ tumor and one ɑ_v_β_3_^-^ tumor representative of three others, 24 h after Angiostamp™ 700 i.v. injection. Scale bars represent 1 cm. **(C, D)** immunohistochemistry directed against ɑ_v_β_3_ integrins to confirm the ɑ_v_β_3_ status of the tumors. Scale bars represent 200μm.

Immunohistochemical examination confirmed the α_v_β_3_ integrin status of tumors (Figure 1C and 1D). The α_v_β_3_-positive tumors exhibited a strong labeling (Figure 1C), while blood vessels (arrow) acted as positive controls for α_v_β_3_-negative tumors.

### Specificity of Angiostamp™ targeting

Integrins are known to be expressed on the surface of endothelial cells of blood vessels, and tumors are characterized by a strong neoangiogenesis. Because Angiostamp™ was fixed to non-α_v_β_3_-expressing tumor cells, we assessed whether it could label tumor-associated endothelial cells. For this purpose, we performed macroscopic and microscopic fluorescence analysis on the tumor cells and endothelial cells located inside tumor nodes tumor cells and endothelial cells) to locate the Angiostamp™ fixation to the different cells. We used GFP (green fluorescent protein)-expressing tumor cells and fluorescent antibodies against endothelial cells, and analyzed the colocalization of Angiostamp™ and the GFP-expressing tumor cells and/or the labeled endothelial cells. The genetically modified α_v_β_3_-positive ovarian adenocarcinoma cells (SKOV-3) that constitutively expressed eGFP (enhanced GFP) were injected into nude mice. The mice were sacrificed 21 days after the injection of tumor cells, and 18 h post-Angiostamp™ injection. Animals were imaged at a macroscopic level using GFP and Cy5.5 filters and biopsies were observed at the microscopic level using specific labeling (collagenase-4 and CD31) with the appropriate set of filters (Figure 2). This experiment was reproduced in three different mice.

**Figure 2:** Fluorescence imaging of tumor nodules using Angiostamp™ Mice were injected i.p. with 10^7^ eGFP-expressing SKOV-3 cells. After 20 days, mice were injected with Angiostamp™ 700. They were sacrificed 24 h after injection and analyzed after laparotomy. **(A)** Fluorescence macroscopy shows eGFP-expressing tumor cells detected using a GFP filter set (left); Angiostamp™ 700 labeling was detected using Cy5.5 filter set (right). GFP-positive cells were found in the ovary (not shown) and on the surface layer of the uterus and colon (left image). The Angiostamp™ labeling identified the tumor localization (right). **(B)** *Ex vivo* fluorescence microscopy on histological section (x100 objective). Nuclei were labeled with DAPI (blue), eGFP-expressing tumor cells were detected with a GFP filter set (green); autofluorescence in Cy5 is shown (red), and Angiostamp™ 700 was detected with a Cy5.5 filter set (orange). **(C)** Fluorescence microscopy on histological sections (x100 objective) were analyzed after immunostaining performed with anti-collagenase 4 antibodies. Nuclei were labeled with DAPI (blue), eGFP-expressing tumor cells were detected with a GFP filter set (green); anti-collagenase-4 antibodies were labeled with Cy5 (red), and Angiostamp™700 was detected with a Cy5.5 filter set (orange). **(D)** Fluorescence microscopy on histological sections (x100 objective) were analyzed after immunostaining performed using anti-CD31 antibodies. Merged images of two independent tumors are shown. Nuclei were labeled with DAPI (blue), anti-CD31 antibodies labeled with Cy3 (green), and Angiostamp™ 700 was detected with a Cy5.5 filter set (red). Scale bars represent 15μm.

Macroscopic analysis of tumor nodules demonstrated that (Figure 2A) the Angiostamp™ labeling was not as precise as the eGFP labeling. There was not a strong colocalization of the labeling of tumor cells or of other cells, such as endothelial cells. The Angiostamp™ labeling was more diffuse and was not restricted to the tumor location depicted by the eGFP expression, suggesting that other components of the microenvironment contributed to the overall labeling.

Tumor biopsies were then frozen and prepared as described in the Material and Methods. Sample analysis occurred either directly (Figure 2B) after cryosectioning or after immunostaining with anti-collagenase-4 (Figure 2C) or anti-CD31 (Figure 2D) antibodies to visualize endothelial cells (vessels) using fluorescence microscopy. We observed an inhomogeneous staining corresponding to Angiostamp™ inside some but not all tumor cells (Figure 2B). The colocalization of eGFP and Cy5.5 staining was not as strong as expected, but the results confirmed that Angiostamp™ was interacting with some but not all tumor cells.

We next performed immunostaining to visualize other components of the tumor, namely the vessels, using anti-collagenase-4 (Figure 2C) and anti-CD31 (Figure 2D) antibodies in combination with Angiostamp™ staining. As observed in Figure 2C, Angiostamp™ did not particularly stain vessels even though we were sure of the αvβ3 expression, as we were for the SKOV-3 tumor cells (Figure 1D). Angiostamp™ 700 labeling was more restricted to the tumor cells; this was confirmed using anti-CD31 antibodies. We observed a diffuse colocalization between Angiostamp™ 700 labeling and tumor vessels (Figure 2D).

The fact that Angiostamp™ could label tumors irrespective of their α_v_β_3_ integrin status, and that co-staining of Angiostamp™ and tumor cells revealed greater tissue labeling than could be explained simply by staining of neoangiogenesis, led us to hypothesize that the “enhanced permeability and retention” (EPR) phenomenon could be implicated. Indeed, EPR plays an important role for passive targeting to tumor tissues, by allowing greater entrance of drugs or probes due to the endothelial cell fenestrations that occur in angiogenic tumor vessels. Angiostamp™ could then be internalized by tumor cells, regardless of their α_v_β_3_ integrin status.

### Broader utilization of Angiostamp™ for tumor detection

These observations led us to propose a broader use of Angiostamp™ for tumor detection regardless of the tumor expression of α_v_β_3_ integrins. We injected nude mice subcutaneously (s.c.) with 10^7^ human tumor cells from different origins. We used: ovarian adenocarcinoma cells (SKOV-3) [20], glioma cells (U87) [22], and colorectal carcinoma cells (HCT 116), all expressing high levels of integrins (Figure 3A); head and neck carcinoma cells (CAL33) [21], breast carcinoma cells (SKBR3) [22]), and human ovarian adenocarcinoma cells (HOAC) (OVCAR) [23], all expressing medium levels of integrins (Figure 3B); and breast carcinoma cells (MDA-MB 231) [24], expressing low levels of integrins (Figure 3C). Each cell type was injected into two animals in two different and independent experiments, in accordance with the ethical use guidance for animal models. Cells were allowed to grow *in vivo* for three weeks, and tumor nodules that developed were imaged without surgery. The use of Angiostamp™ resulted in successful imaging of all tumor types in all animals, including both high-α_v_β_3-_expressing and low-α_v_β_3_-expressing tumors, although we detected different levels of fluorescence intensities. For high levels of integrin expression (Figure 3A), mean tumor fluorescence intensities were >15 AU (defined as the fold increase from the background, arbitrary units) (17, 21.4, and 16 AU for SKOV-3, U87, and HCT-116, respectively), for medium levels of integrin expression (Figure 3B), mean tumor fluorescence intensities were around 8 AU (8.1, 8.2, and 8.6 AU for CAL33, SKBR3, and OVCAR, respectively), and for low levels of integrin expression (Figure 3C), mean tumor fluorescence intensity was 3.4 AU for MDA-MB 231. As previously stated, for quantification we used as a background value the brightest part of the image adjacent to the tumor.

**Figure 3:** Angiostamp™ clearly depicts different tumor nodules whether or not they express ɑ_v_β_3_ integrins *In vivo* real-time fluorescence images of **(A)** nodules from s.c. injection of ovarian adenocarcinoma cells SKOV-3, glioma cells U87, or colorectal carcinoma (HCT116 cells). **(B)** nodules from s.c. injection of head and neck cancer cells CAL33, breast carcinoma cells SKBR3, and ovarian adenocarcinoma cells OVCAR-3. **(C)** nodules from s.c. injection of breast carcinoma cells MDA231 **(D)** detection of tumor dissemination in ascite-bearing mice, following i.p. injection of ovarian adenocarcinoma SKOV-3 cells, OVCAR-3 cells, or cells or colorectal origin (HCT116 cells). Live mice were analyzed. For each cell type, one mouse is presented that is representative of two experiments in total.

We also used Angiostamp™ to evaluate the tumor dissemination of peritoneal cancer cells in live animals with ascites, without the use of surgery, by imaging ascites-bearing mice (after intraperitoneal (i.p.) injection of SKOV-3, OVCAR-3, or HCT116 cells (Figure 3D). The technique detected tumor progression despite a substantial ascite volume.

We therefore conclude that, following either s.c. or i.p. injection of tumor cells, Angiostamp™ is a powerful tracer to visualize all tumor nodules irrespective of their α_v_β_3_ integrin status.

### Kinetic analysis of Angiostamp™ fixation

In all previous experiments, we injected 2 nmol of Angiostamp™ and analyzed the mice 18–24 h post-injection. Because of nonspecific targeting to the bladder or kidneys, before using Angiostamp™ in pets we performed a kinetic analysis of the signal, from 1 h to 48 h, to ensure the best signal/background ratio. Mice received 10^7^ SKOV-3 cells (human ovarian adenocarcinoma cells) either i.p. or s.c.. Twenty-one days later, we injected mice with Angiostamp™ and analyzed the fluorescence intensities using a Fluobeam^**®**^ camera. This experiment was performed three time (three different mice). Results are presented in Figure 4. The skin of the tail was fluorescent 10 mins after the intravenous (i.v.) injection. After 10 mins, the signal exponentially decreased. Kidneys were rapidly fluorescent (within 1 h) and the fluorescence then decreased rapidly to stabilize at 5 h post-injection.

**Figure 4:** Kinetic analysis of Angiostamp™ fixation The relative fluorescence intensities for the tumor and the elimination organs (bladder and kidney) were plotted as a function of time. The fluorescence was relative to the skin or the adjacent organ.

The probes accumulated in the bladder at 2 h 30 post-injection. The fluorescence decreased after 3 h to reach a basal fluorescence level at 5 h post-injection. The best ratio of tumor-specific fluorescence/background was obtained between 17 h 30 post-injection and 24 h post-injection (adjacent organ was used as background). After 17 h 30, fluorescence was stabilized in all organs concerned (tumor, bladder, kidneys) and then slowly decreased after 24 h (not shown). Fluorescence could be visualized until 5 days post-Angiostamp™ injection. We selected 17 h 30 as the time point for further investigations, as at this time point we were able to visualize a high intensity of fluorescence in tumor nodules whether cells had been injected s.c. or i.p..

### Guided surgery with Angiostamp™/Fluobeam^®^ in pets

The Angiostamp™/Fluobeam^**®**^ technology required testing for its utility in helping surgeons visualize tumor nodules during surgery. For this purpose, we initiated a proof of concept trial on pets. Here, we report four veterinary cases: one cat and three dogs bearing different tumor types (breast and ovarian cancer). All of them received a single injection of Angiostamp**™** the day before surgery (between 15–18 h before surgery) at the dose of 0.15 mg/kg for dogs and 0.3 mg/kg for the cat. The injected dose of Angiostamp™ was determined by the manufacturer.

Animals were anesthetized using ketamine/isoflurane; anesthesia was maintained for the entire duration of the surgery. They stayed for observation for one night in the veterinary clinic, where they received treatment for pain related to surgery. They were returned to their owners the following day with a prescription for pain relief. One (case N°4) received anticancer treatment (platinum salt) after the surgery because of ovarian cancer dissemination.

#### Case N°1

A female cat presented with palpable masses on mammary glands. The biggest mass measured 5 cm^3^ and required removal (Figure 5A). The veterinary surgeon wanted to determine whether an additional palpable smaller nodule (Figure 5E) was associated with the biggest mass, and whether it was cancerous. We observed the nodules with Fluobeam^**®**^ before (Figure 5B and 5F) and after their removal (Figure 5C and 5G, *ex vivo* imaging).

**Figure 5:** Angiostamp™ allowed visualization of mammary carcinoma as well as the draining lymph nodes **(A)** The cat had a single visible tumor. **(B)** *In vivo* real-time fluorescence images of the tumor nodule before and **(C)** after resection. **(D)** Pathological analysis revealed the carcinoma component of the tumor. **(E)** There was no evidence of other visible tumor. **(F)** *In vivo* real-time fluorescence images revealed fluorescent draining lymph nodes before **(G)** and after resection. **(H)** Pathological analysis revealed the carcinoma component of the draining lymph nodes.

Both nodules were labeled with Angiostamp™, with differing intensities. The biggest mass was positive with an intensity of fluorescence of 8 AU (compared to the adjacent skin). Pathological analysis revealed a malignant carcinomatous tumor with heterogeneous aspects (Figure 5D). The smaller nodule was less fluorescent (5 AU, compared to the adjacent skin). The veterinary surgeon decided this required removal because of previous data stating that a fluorescence intensity above 3 AU indicated abnormal cells. Pathological analysis revealed an adenomatous hyperplastic mammary gland without carcinomatous signs (Figure 5H). All of the lymph node chain (not shown) exhibited varying fluorescence intensities (around 5 AU).

In this case, Angiostamp™ allowed the surgeon to visualize different nodules during surgery and to decide whether they required removal. Pathological analysis confirmed that the biggest nodule was cancerous and revealed that the second was hyperplasic. The other positive nodules corresponded to the entire lymph node chain; in this case, they were not removed.

#### Case N°2

A female dog presented with two nodules on mammary glands possibly requiring removal; veterinary surgeons wished to determine whether the nodules were cancerous or not. The dog was injected with Angiostamp™ and the nodules were analyzed the following day with Fluobeam^**®**^ before their biopsy. The nodules proved negative for Angiostamp™ labeling and biopsy revealed they were free of tumor cells (not shown).

In this case, the dog also had a nodule on the sternum (Figure 6A) that the surgeon expected to be benign. However, we analyzed it with Fluobeam^**®**^ and found that it was labeled with Angiostamp™ (Figure 6B, fluorescence intensity >3 AU). It was removed and analyzed by a pathologist, who determined that the nodule was a carcinomatous extension of a cutaneous tumor (arrow) between the pilosebaceous units (^*^) (Figure 6C). To summarize, in this case we deliberated whether nodules on mammary glands required removal, and fluorescence imaging indicated that the glands were normal. Pathological analysis confirmed there was no malignancy. The dog presented with another nodule expected to be benign. However, it was labeled with Angiostamp™, and was in fact shown to be a tumor (Figure 6B, 6C).

**Figure 6:** Angiostamp™ allowed intraoperative detection of a canine carcinomatous extension cutaneous tumor **(A)** The dog displayed only one nodule, which was expected to be benign. **(B)** *In vivo* real-time fluorescence images of the nodule. **(C)** Pathological analysis revealed a carcinomatous extension of a cutaneous tumor.

#### Case N°3

A 10-year-old female French bulldog presented with suspected ovarian cancer in one ovary. The owner wanted the surgeon to verify that the tumor had not metastasized and requested that the ovary be removed if it had not. The dog received Angiostamp™ 18 h before surgery. We performed imaging on the whole peritoneum after incision (Figure 7A and 7C). This imaging procedure took about 10 mins. We observed that the first ovary was labeled with Angiostamp™ (mean fluorescence intensity of 3.AU, Figure 7D compared to the adjacent organ). The second ovary was also positive (Figure 7E), as well as part of the colon (mean fluorescence intensity of 4 AU Figure 7F). We decided to remove the two ovaries and part of the colon. The surgeon was able to remove all the tumors, and the dog was returned to its owner the following day.

**Figure 7:** Angiostamp™ allowed intraoperative detection of a canine ovarian carcinoma and peritoneal carcinomatosis **(A)** The dog had an ovarian carcinoma in one ovary. **(B)** *In vivo* real-time fluorescence images of the peritoneum. **(C)** There was no visual sign of carcinogenesis. **(D)** *In vivo* real-time fluorescence images of the right and **(E)** the left ovary, as well as **(F)** the colon. **(G)** and **(H)** pathological analysis revealed carcinoma of the papillary predominant architecture, with cribriform and glandular architecture on the two ovaries. **(I)** Carcinomatous infiltration of the muscular and serous layers of the part of colon resection.

Pathological analysis revealed that both ovaries contained tumor cells. Figure 7G shows carcinoma of the papillary predominant architecture, with cribriform and glandular architecture, and Figure 7I shows carcinomatous infiltration of the muscular and serous layers of the digestive resection. The colon contained external carcinomatous infiltrations of the bowel (arrows).

#### Case N°4

A 13-year-old Maltese dog presented with suspected ovarian cancer in one ovary, which was thought to have disseminated. The dog received Angiostamp™ 24 h before surgery. The whole peritoneum was analyzed first without fluorescence and then with Fluobeam®. The entire procedure took about 15 mins. Without fluorescence imaging, there was good evidence that the colon contained tumor nodules (Figure 8A). Detection of Angiostamp™ labeling confirmed this (Figure 8B) (mean fluorescence intensity of 5 AU in the colon). When we examined the peritoneum as a whole with fluorescence imaging, the surgeon was unable to detect nodules (Figure 8E), but fluorescence emissions were found in the liver (Figure 8F) and in the uterus (Figure 8J) (mean fluorescence intensity of 5AU in the uterus). As in case N^o^3, we performed imaging on the first ovary at the beginning of the laparotomy and found that it was labeled with Angiostamp™ (mean fluorescence intensity of 13 AU Figure 8C). The second ovary was also positive (mean fluorescence intensity of 11AU, Figure 8G), despite the surgeon’s original view that this ovary did not contain tumor nodules. It was removed, along with the uterus. Other organs were not removed in order to keep the dog alive, according to the owner’s wishes. In parallel, as in case N^o^2, when we examined the anesthetized dog before surgery, we observed two small nodules on the mammary glands. These nodules were removed as they were labeled with Angiostamp™, with a fluorescence intensity of 8 AU on the main tumor (compared to the adjacent skin) and 5 AU for the metastatic point on the adjacent nodule (Figure 8K). The dog was returned to its owner the following day. Because of the metastatic spread visualized with fluorescence imaging during surgery, the dog received chemotherapy treatment two weeks after surgery.

**Figure 8:** Veterinary clinical trial of fluorescence molecular imaging-guided surgery using Angiostamp™ in a case of disseminated canine ovarian cancer **(A)** Color image of the abdominal cavity of the colon and **(E)** the liver. **(B)** Fluorescence image of the abdominal cavity (same area as in A) and **(F)** same area as in E. **(C)** Tumor-specific fluorescence image of the right and **(G)** of the left ovary. **(I)** and **(J)** uterine tract. **(K)** Fluorescence image of two small nodules on the mammary glands. **(D)** Pathological analysis of the right and **(H)** the left ovary. **(L)** Pathological analysis of a mixed mammary tumor with a benign adenomatous component and a benign chondromatous component.

Pathological analysis revealed that both ovaries contained tumor cells (Figure 8D and 8H), as did the uterus. Likewise, the mammary gland nodule contained carcinoma cells (Figure 8L). This mixed mammary tumor also exhibited a benign adenomatous component and a benign chondromatous component.

These data demonstrate that intraoperative tumor-specific fluorescence imaging could improve intraoperative staging and help achieve more radical cytoreductive surgery.

## DISCUSSION

Particularly in cases of carcinomatosis, surgeons need to be able to easily detect tumor cells at various different times. In the case of several peritoneal cancers, at the time of diagnosis, and following physical examination and imaging, an exploratory laparotomy or laparoscopy is usually carried out for histological confirmation and staging. Then, to treat the cancer, the surgeon attempts to remove all visible tumors within the peritoneal cavity, [23] a procedure termed cytoreductive surgery or tumor debulking [24]. For example, in the case of ovarian cancers, surgeons perform a total abdominal hysterectomy, remove ovaries (oophorectomy) and fallopian tubes, and examine all peritoneal surfaces. The surgeons then perform an infragastric omentectomy, pelvic and para-aortic lymphadenectomies, biopsies of clinically uninvolved areas, and extensive peritonectomies, in order to remove as many tumor cells as possible. This sequence of analysis and cytoreductive surgery is also required for other peritoneal cancers, such as colorectal cancer and rare peritoneal diseases, where a precise diagnosis of peritoneal dissemination is also necessary to determine the appropriate treatment strategy. For other tumors that are likely to be non-disseminated, surgery must also be completed with tumor-free margins, and the draining lymph nodes must be evaluated for potential tumor cell invasion. For all these purposes, a technique for imaging tumors that could be performed in intraoperative conditions would be of huge benefit.

Several dyes have previously been tested for clinical use. Indocyanine green (ICG) has been proposed as a good NIR-imaging agent candidate for the detection of peritoneal ovarian tumor nodules [4, 25]. It has been tested for staging in cancer patients [26], and Tummers et al. initiated a trial to determine the feasibility of intraoperative ovarian cancer metastases imaging using NIR fluorescence imaging and ICG in a clinical setting. These authors concluded that, despite detection of all malignant lesions, the high false-positive rate observed highlights the need for a tumor-specific intraoperative agent [27]. As the specificity of fluorescent probes could be enhanced by combining them with a molecular targeting agent, several compounds have been suggested. Bahmani et al. constructed polymeric nanostructured particles loaded with ICG and functionalized with monoclonal antibodies directed against the HER2 receptor. They proved the efficacy of this approach in intraoperative detection and imaging in murine models [4], and will soon evaluate their compound in a clinical setting.

The fluorescent dye 5-ALA is an intermediate substrate of heme metabolism. The administration of 5-ALA to patients results in tumor-specific accumulation of protoporphyrin IX (PpIX), which emits red fluorescence with blue-light irradiation. It is currently used for fluorescence-guided resections of several tumors, such as high-grade gliomas, ovarian cancers [28], superficial bladder cancer, or colorectal metastasis. For this purpose Kondo et al. administered 5-ALA orally to patients 3 h before surgery. The abdominal cavity was observed under light and fluorescence. In one patient, a small fat lesion that was missed under white light observation was detected by ALA-induced fluorescence and was pathologically diagnosed as peritoneal metastasis [6]. The authors concluded that 5-ALA and photodynamic diagnosis is a promising candidate for diagnosing peritoneal dissemination of cancer, but that there are still the issues of undesirable accumulation of PpIX and autofluorescence of the surrounding tissues that require elimination to allow better contrast [6].

Alexander et al. used activatable galactosyl human serum albumin (hGCA)-fluorophore pairs to target lectin receptors expressed on ovarian cancer cells. They concluded, as had the previous authors, that their dye (hGCA-NMP1 in this case) is useful in imaging peritoneal ovarian cancer dissemination both superficially and deep in the abdominal cavity [29]. The limitation of these agents is the fact that they detect only 75% of all lesions, meaning that the technique requires improvement. Moreover, the presence of hemorrhagic ascites greatly reduces the rate of detection [30].

The particular intraoperative NIR imaging that we used in this publication (Fluobeam^®^) has been shown to have many clinical applications. It can be used for parathyroid gland detection using autofluorescence imaging [31, 32]. In breast reconstruction, ICG visualized with Fluobeam^®^ can be used to detect poorly perfused areas of the free flap, evaluate microvascular anastomosis for patency, and assess superficial inferior epigastric artery flap vascular territory for use as an alternative free flap with minimal donor site morbidity [33]. Swanson et al. used Fluobeam^®^ with a 5-ALA-derived component (CLR1502) to detect tumor fluorescence for brain tumor resections (using NIR imaging). This proof of concept study for fluorescence-guided glioma surgery demonstrated high-contrast tumor visualization compatible with surgical applications in mice [34]. Using the same component (CLR1502), Deming et al. showed that intestinal tumors could be analyzed, and that the intensity of the fluorescence signal correlated with the histological characteristics for each tumor. The detection was specific, as colon adenocarcinomas demonstrated increased accumulation of CLR1502 compared to noninvasive lesions. In addition, the authors describe the use of NIR dyes for lymph node analysis and showed that metastatic mesenteric tumors and uninvolved lymph nodes were detected [35]. In the same way, Hirche et al. analyzed the feasibility of the Fluobeam® 800 imaging system in detecting the sentinel lymph nodes using fluorescence retention (using ICG fluorescence imaging). They showed that NIR imaging can be applied to lymphatic imaging for lympatico-reconstructive surgery and sentinel lymph node biopsy [36]. All the compounds described here could enhance the ability to properly remove all tumor cells, through better localization of the primary tumor and improved lymph node identification as well as detection of distant disease.

In this publication, we used a RAFT-c(RGDfK)4-Alexa Fluor 700, which is a fluorescent tumor-targeting probe (Angiostamp™). This compound has previously been used in work by the JC Coll group and ourselves [13, 16, 37]. It was not expected to be specific to tumor cells, as it targets the α_v_β_3_ integrins, which are expressed by endothelial cells. In previous work, however, we showed that Angiostamp™ labeling of tumors was specific. We examined more than 100 mice bearing intraperitoneal disseminated ovarian adenocarcinomas; analysis of fluorescent and nonfluorescent biopsies proved that fluorescence occurs only in the presence of tumor cells. We demonstrated that unless tumor cells were present, we were only able to detect labeling in the kidneys and the eliminatory organs, the uterus for some female mice, and three lymph nodes. Angiostamp™ is therefore a good and specific targeting agent. In order to investigate the potential of Angiostamp™ for widespread clinical use, we investigated whether Angiostamp™ could be used to detect different types of tumors. We showed here that it can target several solid cancers including carcinoma, adenoma, and glioma, from various origins (breast, ovary, colon, brain, lung, head and neck, etc.). In fact, in our evaluation we were able to detect tumor nodules in all mice injected with human tumor cells (data not shown). This was surprising, as current literature suggests that integrins are expressed by only 25% of tumors. As it was initially developed to target tumor angiogenesis (endothelial cells), we investigated whether Angiostamp™ could detect tumors nodules independently of whether or not they express high levels of α_v_β_3_ integrins. We found no correlation between the level of tumor detection and the expression of α_v_β_3_ integrins, suggesting that targeting of integrins related to the tumor-associated neoangiogenesis is sufficient for a good labeling of the tumors by Angiostamp™. In order to prove the labeling of the tumor neovasculature by Angiostamp™, we built a model in which integrin-positive genetically engineered tumor cells or endothelial cells were easily identified by GFP fluorescence or fluorescent antibodies, respectively. Our aim was to demonstrate the colocalization of Angiostamp™ and the GFP-expressing tumor cells, or the colocalization of Angiostamp™ and the antibody-labeled endothelial cells, or both. Macroscopically, we observed a close correlation between Angiostamp™ labeling and GFP expression. Microscopically, we detected Angiostamp™ labeling on some tumor cells, but not all, and on some endothelial cells, but not all. There was no strong association of the dye with all the tumor cells or endothelial cells, suggesting that the Angiostamp™ labeling of tumors could be due to other phenomena. We hypothesize that the EPR effect, which plays an important role in passive targeting to tumor tissues [38]. This phenomenon has been described by Rijcker et al. in 2007, among others [38]. EPR occurs because of disordering in the epithelial cells of tumor tissue, which results in an increased permeation of drugs or probes. Indeed, EPR plays an important role for passive targeting to tumor tissues, by allowing greater entrance of drugs or probes due to the endothelial cell fenestrations that occur in angiogenic tumor vessels. In our experiments, therefore, it may be that, whatever the tumor type, Angiostamp™ is able to cross tumor blood vessels and accumulate in the interstitial tissue.

Importantly, here we were able to visualize all types of tumors tested using Angiostamp™.

Our oncology study in tumor-bearing pet dogs and a cat confirmed that use of the tracer Angiostamp™ and the Fluobeam® camera enabled intraoperative detection of carcinomatosis sites. We examinated unrelated animals requiring treatment for cancer. The intraoperative detection of the animals’ carcinomatosis sites made the surgery easier for the veterinarians (as it aided detection of the tumor nodules, and helped in the decision of whether or not to remove organs, such as ovaries, uterus, etc), and faster. The four veterinarians stated that the technique could be improved by knowing the value of fluorescence above which nodules should be removed in different types of cancer. Here, we used a cut-off fluorescence intensity value of 2 AU; all the nodules removed contained tumor cells. Our results can be assessed alongside those of the study described by Liberale and al. [39], in which these authors performed a clinical trial on 14 patients using free ICG to detect peritoneal metastases due to colorectal cancer. In this trial, all fluorescents nodules were removed whether they exhibited low, moderate, or high fluorescence, and there was no cut-off value for tumor-to-background fluorescence intensity; a total of 53 resected nodules were found to be malignant, but 10 nodules were benign. However, the resection of benign nodules did not affect the outlook of the patients. Using Angiostamp™ and a cut-off value of 2 AU, all the nodules we resected from pets were found to be malignant. The study by Liberale and al. highlights that **intraoperative** fluorescence imaging is of benefit for patients; for four of the 14 patients, the surgery was modified by intraoperative ICG fluorescence imaging that detected metastatic nodules that had not been revealed during standard work-up and surgery. This fits with our observations in pets. The limit of ICG labeling is that it is not efficient for nodules from mucinous tumors. Angiostamp™ appears to have a larger application [13]. Finally, although it is reasonable to think that fluorescence exploration could be poorly informative in patients with advance peritoneal dissemination [39], the majority of patients with either colorectal or ovarian cancers have limited disease with a median PCI score of 8, and so fluorescence imaging could also be used at the time of diagnosis when surgeons perform an exploratory laparotomy or laparoscopy for staging. In conclusion, fluorescence imaging that targets α_v_β_3_ integrins could therefore be an important tool to aid peritoneal exploration and complete resection of tumors, with the added benefits of nontoxicity and good tolerability. Following these important results, a phase I/II study using the Angiostamp™/Fluobeam® fluorescence detection system in peritoneal carcinomatosis will be conducted.

## MATERIALS AND METHODS

### Cell culture

The HOAC line IGROV-1 was provided by the Gustave Roussy Institute [40]. HOAC SKOV-3 cells (ATCC^®^ HTB–77), colon carcinoma cells HCT116 (ATCC^®^ CCL-247), glioma cells U87 (ATCC^®^ HTB-14), head and neck carcinoma cells (CAL 33), and breast adenocarcinoma cells MDA-MB 231 (ATCC^®^ HTB-26) and SKBR3 (ATCC HTB-30) were obtained from the American Type Culture Collection (Manassas, VA). Human melanoma cells (LB319 MEL) were a personal gift from AF Tilkin-Mariamé (France). They were routinely cultured as previously described [41] in RPMI with 10% fetal calf serum. Cell lines were routinely checked for mycoplasma.

SKOV-3 cells were genetically modified with an eGFP coding gene using a lentiviral vector (pWPXLd-1, Trono lab, Switzerland) and selected by flow cytometry for a high and stable expression of eGFP as described previously [19].

### Animal experiments on mice

Female Swiss athymic nude mice, 4–5-weeks-old (Charles River Laboratories, L’Arbresle, France), were housed in filter-capped cages and kept in a sterile facility, which was maintained in accordance with the standards of the Federation of European Laboratory Animal Science Associations in accordance with the AACR statement for the use of animals in cancer research. The Claudius Regaud Institute animal ethics committee approval was obtained for use of the animal model and the study protocols. A two-week quarantine period was imposed on all mice before starting the study. The i.p. and the s.c. injections used to inject ovarian adenocarcinoma cells, as well as glioblastoma, breast, and colon cancer cells, were as described previously [41, 42]. The i.v. tail vein injection of melanoma cells used to generate lung metastasis were described in Pich et al. [43].

### Immunohistochemistry

Tumors were removed and fixed in formalin for 24 h. They were then paraffin embedded. Sections were cut at 4 μm and stained using a hematoxylin and eosin procedure.

To examine the expression of α_v_β_3_ integrins, tumors were removed and fixed in RCL2® (Alphelys™SA, Plaisir, France). Immunohistochemistry was performed as described previously [13] using an antibody against α_v_β_3_ integrins (dilution 1:100 from Millipore).

### Detection of Angiostamp™-targeted cells in ovarian cancer xenografts

At day 0, five mice received i.p. 10^7^ genetically modified GFP-expressing IGROV-1 cells. After 19 days, tumor-bearing animals received 2 nmol of Angiostamp™ 18 h prior to analysis, as specified by the manufacturer. Fluorescence macroscopy was carried out using a “Macrofluo” fluorescence microscope (Leica Microsystems SA, Rueil-Malmaison, France), equipped with a Cool Snap HQ2 Camera (Roper Scientific, Photometrics, Tucson, AZ, USA) at x2 magnification. Tumors were then removed and fixed in 3% paraformaldehyde for 24 h, then 20% sucrose for another 24 h. The tissue was then mounted in optimum cutting temperature (OCT) compound (Tissue-Tek, Sakura Finetek, NL) and frozen at -55°C. Sections of 10 μm thickness were cut from the OCT compound blocks using a cryostat (Leica CM3050 S) at -20°C. DAPI staining in Moviol mounting medium was used for visualization of cell nuclei. Histological sections of tumors were observed under a Leica DMIRB fluorescence microscope (Leica Microsystems) with an x100 oil objective. GFP or Angiostamp™ fluorescence in tumors was detected after selective excitation produced with a compact arc source (Leica Microsystems, Wetzlar) and a GFP filter (λex:480/40; λem:527/30) or Cy5.5 filter (λex:665/45; λem:725/50) (Chroma Technology, Brattleboro, VT). High-resolution 16-bit images of 1392 x 1040 pixels were captured using a cooled charge-coupled device camera (CCD) camera (coolSNAP-HQ2, Roper Scientific) and processed for contrast and brightness using MetaVue 6.2 software (Universal Imaging).

### Intraoperative fluorescence imaging

Tumor tracking was performed with the previously described handheld NIR 2D-fluorescence reflectance imaging device Fluobeam ^®^700 or Fluobeam^®^ 800 (Fluoptics, Grenoble, France) according to the Angiostamp™ labeling used (700 or 800). This system consists of a control unit, with a laser source emitting at 680 or 785nm respectively; the laser beam is then fiber guided from the control unit to the optical head, allowing for a 6-cm spot diameter at a working distance of 17 cm in the field of view, and an optical head consisting of a CCD camera and white light-emitting diodes for the illumination of the field of view. The relative fluorescence intensity is the ratio between the fluorescence intensity of the considered organ and an “internal control”. To quantify the relative intensity, the respective intensity of the skin near to each organ (i.e., near to the tumor or to the elimination organs, the kidneys and bladder) was used as specific internal control.

The fluorescence intensity was evaluated by measuring the mean fluorescence intensity on several selected areas using ImageJ. For each measure, the value of the background signal was subtracted.

### Use of Angiostamp™ in veterinary practice

Client-owned dogs presenting at the veterinary clinic ‘Alliance’ (Bordeaux and dependencies, France) with suspected spontaneous ovarian cancers were prospectively enrolled in this study between July 2012 and July 2014. Tumor diagnosis was performed preoperatively using ultrasound imaging. Other eligibility criteria required that dogs be free of significant co-morbid illness with a favorable performance status. After diagnosis, the owner’s consent was obtained in each case. Data retrieved from the medical records included breed, sex, age, body weight, preoperative diagnosis, and anatomic location of the tumor. Complete clinical staging was performed before surgery. Real-time fluorescence imaging was performed using the compact and portable 2D fluorescence reflectance imaging devices, Fluobeam^®^ 700 or Fluobeam^®^ 800, according to the Angiostamp™ labeling. The Fluobeam^®^ 800 device was used with a dedicated single-use sterile cover bearing an optical window, compatible with NIR fluorescence measurements and with the aseptic conditions of the operating room as described previously by Cabon et al.[44, 45].

Study protocol: All dogs received a single i.v. injection of Angiostamp™ the day before surgery (between 15 and 18 h before surgery), at a dose of 0.15 mg/kg for dogs and 0.3 mg/kg for cats. To calculate the doses required, a table of dose equivalence was used, which is cited in the manufacturer’s “drug or diagnostic agent development guidelines” relating to Angiostamp™. Typically, this table is used to calculate the dose that will eventually be injected into humans, depending on the dose used in animals (in preclinical trials). The factors to be applied are shown by species. The dose that was commonly used in mice was 2 mg/kg, but in an effective dose manipulation, it was seen that this dose could be halved (1 mg/kg). The corrective factor between mice and dogs is 6.66, so dividing 1/6.66 gave a dose of 0.15 mg/kg for dogs. Because of the difference in body surface area between dogs and cats, we chose to inject 0.3 mg/kg in the cat to maintain an equivalent dose.

Animals were anesthetized using ketamine/isoflurane, and anesthesia was maintained for the entire duration of the surgery. All animals stayed for observation in the veterinary clinic for one night, where they received treatment for pain. Pets were considered off study the day after completion of the surgery and were free to receive any additional therapy deemed appropriate by the attending clinician. They were returned to their owners with a prescription for pain relief for pain relating to surgery.

All tumors were submitted to fluorescence acquisition after resection. The tumors were then sent for conventional histological examination. The tumor was placed in neutral-buffered 10% formalin solution for at least 48 h for fixation. Once fixed, the tumors were embedded in paraffin. Four-μm slices obtained from the paraffin blocks were stained with hematoxylin and eosin and were submitted to a classic histopathological evaluation by a pathologist.

All NIR fluorescence data were collected and analyzed using the ImageJ image-analyzing computer program and Microsoft Excel software. The fluorescence intensity values of the tissue of interest was processed as described in [44]. For fluorescence analysis, in cases of wide excision, healthy tissues were defined as part of the surgical bed (the same tissue found in the tumor-free margins), far from the original tumor, and were validated as ‘‘clean’’ tissue following histopathological analysis.
